# The Influence of Sports Dance on the Physical and Mental Development of Contemporary College Students Based on Health Detection

**DOI:** 10.1155/2022/3715150

**Published:** 2022-06-11

**Authors:** Huali Huang

**Affiliations:** Department of Public Sports, Jingchu University of Technology, Jingmen 448000, Hubei, China

## Abstract

The healthy growth of college students is related to the future development of the country and the prosperity of the nation. Under fierce social competition, college students are faced with academic pressure and employment pressure, resulting in the failure to improve their physical and mental health and their low self-acceptance level. Faced with such a situation, it is an important subject to solve the problem of the physical and mental health development of contemporary college students. As a sport that integrates sports and art, sports dance is worthy of in-depth discussion on the physical and mental development of college students. To analyze the impact of sports dance on the physical and mental development of contemporary college students, this paper uses an intelligent health monitoring system to monitor the health status of college students before and after physical dance exercise. It analyzes the influence of sports dance on the physical and mental development of college students from the aspects of cardiorespiratory endurance, muscular endurance, flexibility, and happiness. Finally, the results are obtained by conducting experiments with 10 college students. The experimental results show that the psychological well-being of college students who take physical dance exercise increases by 7.8%. Cardiorespiratory endurance and flexibility are both improved accordingly. Physical dance exercise promotes the physical and mental development of contemporary college students.

## 1. Introduction

With the progress of human beings and the continuous development of social economy, college education pays increasingly attention to the overall improvement of students' personal quality. In the education of colleges and universities, the physical and mental health and artistic development of students have become essential. The healthy development of students' physical and mental health has become an integral part of the quality education system. With the progress of human beings and the continuous development of social economy, higher education pays increasingly attention to the overall improvement of students' personal quality. In higher education, the physical and mental health and artistic development of students become essential. Students' mental health has become an integral part of the quality education system. College students face enormous pressure in academic, economic, interpersonal, and other aspects, and are prone to psychological barriers and emotional overload due to excessive pressure. Practicing sports dance in colleges and universities can effectively relieve students' stress, regulate their emotions, and reduce the occurrence of extreme mental states. Physical dance exercise can improve the quality of students, but also affect the physical health of college students. Physical dance teaching is closely related to the development of students' mental health. It can promote the improvement of college students' mental health and also plays an important role in the overall development of students' quality.

To promote the development of sports dance, a large number of researchers are devoted to the study of physical health. To study the effect of sports dance on the body shape of young men, C Lu chose young men as the subject of sports dance training. Through training, it is found that the physical fitness of sports men is significantly improved [1]. SJ Zhang studied peripheral blood T cells of retired employees through dance experiments. It was found that the immune function of the elderly who exercised physical dance improved better [2]. HU Mi studied the effect of body dance on the balance ability of girls aged 6 to 7 years and trained the test group for 4 months. The results show that sports dance can significantly improve the static balance ability of girls aged 6 to 7 years [3]. Z Zhang studied the effect of physical dance on the body shape of overweight and obese elderly women through experimental methods, mathematical calculations, and comparisons. After 10 weeks of regular exercise and dancing, it was found that the subcutaneous fat in women was reduced, and the fat accumulation in the waist and abdomen was significantly improved [4]. R Wang studied the effects of participating in competitive dance training on the development of coordination and sensitivity in college students. The results show that sports dance can effectively improve the coordination and sensitivity of ordinary college students [5]. XF Zong has examined changes in college students' physical health through sports and dance programs. The results showed that the teaching and tutoring of a sports dance classes promoted the improvement of students' body shape, physique, physical function, and body balance [6]. MH Gao analyzed the comprehensive level requirements of sports dance coaches in the process of cultivating athletes from three aspects: professional skills, training level, and comprehensive management. It can enhance the ability of coaches to cultivate athletes, to cultivate excellent athletes [7]. These studies show that physical activity plays an important role in people's health. Although these studies have achieved rich results, with the emergence of new technologies and new situations, many college students have new psychological problems, and it is necessary to pay more attention to the psychological research of college students.

Physical dance exercise can not only help people have a healthy body but also promote the development of people's mental health. H. Sun believed that sports dance has become mainstream in sports. It examined the influence of sports dance practice on students' temperaments from aspects of participants' temperament and body shape, personal expression, and self-confidence in sports [8]. Q Lit found that good posture and gait rhythm can be created for adolescents through physical dance practice [9]. JiYoung conducted a three-month study of college students. The study found that exercise changed physical fitness, weight, and psychological values. Sports dance has a positive effect on women's physical health [10]. XB Dong had given extensive physical dance training to more than 200 physical education students. It is found that sports dance can improve the quality, self-esteem, self-confidence, and interpersonal skills of college students [11]. JH Zhu trained the students in gymnastics. It is found that physical dance teaching improves students' “aesthetic quality,” reduces negative emotions, and promotes students' physical and mental health [12]. Using bibliography and comprehensive analysis methods, J. Yao discussed the role of sports dance in cultivating students' healthy beauty, athletic beauty, and shaping physical beauty. It promotes the cultivation of college students' aesthetic ability, creates beauty, and influences the work of aesthetic education [13]. T Cheng conducted a survey of children aged 9–12. Combining questionnaires and mathematical statistics with the Eysenck Children's Personality Questionnaire and a questionnaire tool, it was found that children who had learned sports dance were in better physical condition than children who had not learned sports dance. And their character is more optimistic and upward [14]. The above studies show that sports dance promotes the development of human mental health.

Dance Sports is a perfect combination of art and sports, an activity that includes dance, movement, and music. It has a variety of values such as sports, competition, aesthetics, and fitness and can achieve the purposes of entertainment, competition, and exercise. In this paper, the intelligent health tracking system is used to collect various physical fitness indicators of students in the process of sports dance training and send them to the database wirelessly. After the training, the physical, and mental indicators of the students were collected and compared with those before the experiment to observe the impact of physical and dance exercise on the physical and mental development of college students.

The innovations of this paper are as follows:

1. This paper analyzes the importance of sports dance. It uses an intelligent health detection system to collect student physiological data to analyze the impact of sports dance on students.
2. According to the age and gender of college students, this paper is tested under the same conditions. Each student's level of mental ability is analyzed and some indications of the impact of different physical activity programmes on mental health are provided.
3. This paper uses the intelligent health detection system to study the impact of sports dance on the physical and mental health of students. It improves the effectiveness of data analysis, ensures the accuracy of data, and lays a new foundation for future research.

## 2. Intelligent Health Detection System

### 2.1. Collection of Sports Dance Information

This paper consists of four main parts: the main controller state search module, the remote control module, the smartphone software monitoring module, and the remote monitoring server module. The whole system is shown in Figure 1. The main controller mainly includes three sensing sensors: an oxygen sensing sensor for oxygen collection, diastolic pressure sensors, and a systolic pressure sensor for blood pressure measurement. The remote control unit cooperates with some external auxiliary tools to first record the physical data and parameter data obtained from the sensor. The physical data and parametric data collected by the physical sensors are then transmitted. The unit is monitored via WiFi transmission to smartphone software. The wireless WIFI module used to transmit data to the smartphone monitoring module adopts the serial port-Ethernet-wireless network function. Smartphone software monitoring involves partly managing user information and partly collecting normal student data [15]. The remote monitoring server platform is the same as the computer side. A Tomcat server specially designed for the Internet is installed on the computer. It is used to identify users using remote browsers and to record the physical activity of college students.

### 2.2. Android System

The Android system is divided into upper and lower layers. The upper layer has the application system layer and the application layer, and the lower layer has the kernel layer and the runtime system layer. The Android system architecture is shown in Figure 2. The basic Android server for the Linux kernel layer is called Linux Kernel Layer. It is based on Linux2.6, supports basic functions in Android, and is a movable layer that distinguishes software and hardware. Android kernel libraries are Android components provided by some core libraries. Developers can use it through the application process. Android time zone is configured by Android using Java language. To operate an Android application successfully, it needs to run in the Dalvik virtual machine. The Dalvik virtual machine must be run to run Android applications. The Dalvik virtual machine is a registry-based Linux kernel that provides basic functionality. The Android application framework can provide developers with any API framework they want to use. These technologies enable developers to better develop new applications, such as use of application resources, access to location information, and alarm settings. An Android application is a visual record of Android programming. It includes many source files of Java objects and finally starts the apk package for fetching [16, 17]. Android itself provides many basic applications such as Home, Contacts, Phone, and Browser. At the same time, developers can also use LayerLayerAPI to implement their own programs.

### 2.3. WiFi Wireless Transmission Technology

WiFi is a trade name in the industry. WiFi allows terminals to connect to the Internet anytime and anywhere, which is very convenient for human use. Like wireless technology, WiFi is a technology that can connect wireless devices such as computers, smartphones, and iPads. When using a wireless network, it should be noted that both the Infant network and the ad hoc network belong to the wireless network. The location of the wireless AP network can create a wireless network, making it the central part of the network [18]. Any of these sites (computers, PDAs, and other Internet-enabled user devices) that are connected to a wireless network can be referred to as a site. As the center of the entire network, the wireless AP needs to communicate with other applications. Many STA devices are built in to create these wireless networks, while basic AP-based wireless networks are created by APs [19]. The basic network topology is shown in Figure 3. An ad hoc wireless network is a loose network. The AP is not in the network and only consists of two or more STAs, each of which can communicate with the outside world directly. The effect that the system wants to achieve in this paper is that the smartphone or PC can use WiFi connection to receive the physiological parameter information of college students and combine the data obtained from the home wireless network.

### 2.4. Gateway Workflow

The collection and transmission process of real sports dance training data needs to open the gateway and connect to the Internet. It uses the device to collect dance training data before and after the experiment. Different devices can have different transmission methods, for example, ECG first receives ECG data and then sends data through Bluetooth. The oximeter turns on Bluetooth before uploading data. After the data transmission is completed, the device will wait at the gateway port until it starts to search for data transmission. When the gateway is in standby mode (the delay may be in voting mode), the target Bluetooth device initiates a data request [20]. The device transmits the movement dance data received from the portal. After detecting the end of the data transfer, the Bluetooth is finally turned off. After the gateway analyzes and filters the received data, it processes the data packet of the data path and sends it to the data communication server through the data transmission model. If the gateway device is not connected to the network, the collected data is sorted and stored in a local file, and the data is resent after connecting to the network [21]. The workflow of the gateway is shown in Figure 4.

## 3. Recommendation Algorithm

The focus of this study is to detect videos of college students' physical dance exercises. It uses the intelligent detection system to collect various physical indicators of college students during physical dance exercise and collects exercise videos. In a sequence of video images, the extracted images are simplified and sampled.

### 3.1. Active Contour Tracking Method

The moving edge function can provide target information about the moving position and moving shape of the object. The active contour algorithm is a common algorithm based on tracking edge information [22]. The contour model is an efficient segmentation and monitoring tool that requires parameters to render contours.

(1) $$\begin{array}{c} v\left(s\right)=\left[x\left(s\right),y\left(s\right)\right]. \end{array}$$

The energy of the contour line is defined as

(2) $$\begin{array}{c} E_{a}\left[v\left(s\right)\right]=E_{b}\left[v\left(s\right)\right]+E_{c}\left[v\left(s\right)\right]+E_{d}\left[v\left(s\right)\right]. \end{array}$$

In the formula, *E*_*b*_ represents the internal energy of the active contour, *E*_*c*_ represents the energy of the image force, and *E*_*a*_ represents the energy generated by the external restraint force. Then, the edge detection can get the contour edge of the image. Edge detection can be done by convolution with the help of gradient operators. It can be represented as a vector in position:

(3) $$\begin{array}{c} \nabla f\left(x,y\right)={\left[G_{x}G_{y}\right]}^{T}={\left[\frac{\partial f}{\partial x}\frac{\partial f}{\partial y}\right]}^{T}. \end{array}$$

The direction of the vector is

(4) $$\begin{array}{c} \text{mag}\left(\nabla f\right)={\left[G_{x}^{2}+G_{y}^{2}\right]}^{1/2}. \end{array}$$

### 3.2. Optimal Bayesian Estimation

The mathematical model of the dynamic time-varying system can be described by formula (5) and formula (6). The state update equation of the system is described by

(5) $$\begin{array}{c} x_{a}=f_{a}\left(x_{a-1},v_{a-1}\right). \end{array}$$

Among them, *f*_*a*_ is a nonlinear function of the system state *x*_*a*−1_, and *v*_*a*−1_ is a stationary noise sequence.

The measurement formula of the system is

(6) $$\begin{array}{c} z_{a}=h_{a}\left(x_{a},n_{a}\right). \end{array}$$

Among them, *h*_*a*_ is a nonlinear function of the system state *x*_*a*_ and *n*_*k*_ is a stationary noise sequence.

The basic idea of the Bayesian optimal filtering algorithm is that if the probability function of the initial condition is known, all measurement information can be used to construct the probability function behind the condition. Therefore, any filtering can lead to the theoretical optimal estimate [23]. In mathematical language, it can be described as follows:

(7) $$\begin{array}{c} p\left(x_{a}|z_{1:a-1}\right)=\int p\left(x_{a}|x_{a-1}\right)p\left(x_{a-1}|z_{1:a-1}\right)\text{d}x_{a-1}, \end{array}$$

The state update formula is

(8) $$\begin{array}{c} p\left(x_{a}|z_{1:a}\right)=\frac{p\left(z_{a}|x_{a}\right)p\left(x_{a}|z_{1:a-1}\right)}{p\left(z_{a}|z_{1:a-1}\right)}. \end{array}$$

That is,

(9) $$\begin{array}{c} p\left(z_{a}|z_{1:a-1}\right)=\int p\left(z_{a}{|x}_{a}\right)p\left(x_{a}|z_{1:a-1}\right)\text{d}x_{a}. \end{array}$$

It can be seen from formula (7) that the predictable probability weights can be obtained from the state transition function of formula (5). The probability function can be derived from the measurement model of formula (6). In formula (8), the measured value can be used to change the prepredicted probability to obtain the current state step.

### 3.3. Sequential Importance Sampling

The Bayesian sampling method mentioned above is a simple and commonly used Monte Carlo method. However, it is difficult to calculate over time. The main reason is that every time a desired observation is calculated, a new observation will appear. And the base density needs to be recalculated for each case. To address this issue, the next important sampling idea is proposed. That is, the specific gravity is calculated in the form of regression without changing the sampling time to the previous set of peaks [24].

The purpose of the sampling process is to find the frequency value of a specific sample. The main function must be written as follows:

(10) $$\begin{array}{c} q\left(x_{0:a}|z_{1:a}\right)=q\left(x_{0}\right)\prod_{b=1}^{a}q\left(x_{b}|x_{0:b-1},z_{1:b}\right). \end{array}$$

It can be concluded that

(11) $$\begin{array}{c} p\left(x_{0,a}\right)=p\left(x_{0}\right)\prod_{b=1}^{a}p\left(x_{b}|x_{b-1}\right). \end{array}$$

That is,

(12) $$\begin{array}{c} p\left(z_{1:a}|x_{0:a}\right)=\prod_{b=1}^{a}p\left(z_{b}|z_{b-1}\right). \end{array}$$

It is brought in to get the weight recursion formula:

(13) $$\begin{array}{c} w_{a}=\frac{p\left(z_{1:a}|x_{0:a}\right)p\left(x_{0:a}\right)}{q\left(x_{a}|x_{0:a-1},z_{1:a}\right)q\left(x_{0:a-1}|z_{1:a}\right)}. \end{array}$$

Reconsidering the described Bayesian estimation problem, using the sequential resampling idea, a complete recursive SIS can be obtained. From the point of view of practical application, most literature adopt the idea of sequential resampling. At this point it can be rewritten as follows:

(14) $$\begin{array}{c} w_{a}=w_{a-1}p\left(z_{a}|x_{a}\right). \end{array}$$

Since the main function does not consider the latest data, the model produced by the main function is very different from the model created by the actual background distribution. Especially when the probability function has a probability type, the state setting density or model observations and precision are high. As shown in Figure 5, the sample becomes unusable due to its low density, making this sampling method inefficient.

### 3.4. Particle Scarcity and Resampling

The sampling process is an important part of particle filtering. While it increases particle hunger, it also reduces particle diversity. Therefore, the selection of evaluation should be based on certain criteria [25]. Currently, the most commonly used measurement is based on the number of active particles, defined as

(15) $$\begin{array}{c} N_{f}=\frac{1}{\sum_{i=1}^{N}{\left(w_{t}^{\left(i\right)}\right)}^{2}}. \end{array}$$

The central idea of the particle filter algorithm is to use a random sampling system to represent the desired probability density function rather than based on general states.  Figure 6 illustrates the implementation process of the particle filter algorithm.

The specific implementation steps of the particle filter algorithm are as follows:

(16) $$\begin{array}{c} w_{a}^{\left(i\right)}=w_{a-1}^{\left(i\right)}\frac{p\left(z_{a}|x_{a}^{\left(i\right)}p\left(\right)x_{a}^{\left(i\right)}|x_{a-1}^{\left(i\right)}\right)}{q\left(x_{a}^{\left(i\right)}|x_{0:a-1}^{\left(i\right)},z_{1-a}\right)}. \end{array}$$

If a one-step transition posterior state distribution is used, the formula can be simplified to

(17) $$\begin{array}{c} w_{a}^{\left(i\right)}=w_{a-1}^{\left(i\right)}p\left(z_{a}|x_{a}^{\left(i\right)}\right). \end{array}$$

The normalized weights are

(18) $$\begin{array}{c} {\overset{⌢}{w}}_{a}^{\left(i\right)}=\frac{w_{a}^{\left(i\right)}}{\sum_{b=1}^{N}w_{a}^{\left(b\right)}}. \end{array}$$

The output of the algorithm is the particle set, which is used to approximate the posterior probability and the expectation of the function:

(19) $$\begin{array}{c} \hat{p}\left(x_{0:a}|z_{1:a}\right)=\frac{1}{N}\sum_{i=1}^{N}\delta_{x_{0:a}^{\left(i\right)}}\left(\text{d}x_{0:k}\right). \end{array}$$

That is,

(20) $$\begin{array}{c} E\left(g_{a}\left(x_{0:a}\right)\right)=\frac{1}{N}\sum_{i=1}^{N}g_{a}\left(x_{0:a}^{i}\right). \end{array}$$

## 4. Sports Dance Training Experiment

### 4.1. Experimental Design

Because the research design of this paper is carried out under natural conditions, it does not affect the students' class, and the students do not know the specific experiment, so it has good reliability and validity. It is often used in sports research. The subject and content of sports research often limits the practical application of this rigorous experimental design in many ways. This experimental model is a plan of equal groups before and after the test.

Combined with the research purpose of this paper, this experiment will randomly select from two universities. Students from different majors were randomly selected for the experiment and divided into an experimental group and a control group. Then, the two groups of students were measured with the mental health scale before receiving the experimental training, and the data were recorded. The experimental group was given physical dance exercise for up to 15 weeks, while the control group continued to live a normal life. After the experiment, the experimental group and the control group were remeasured. Finally, the two groups of outcome indicators were statistically analyzed.

### 4.2. Experimental Data

Students of different majors were selected as research subjects. Study and train in a 15-week sports dance class. The control group did not receive physical dance training, but only regularly studied and practiced, while the experimental group received physical dance training. To avoid the interference of age factors, this paper mainly selects sophomore students as the research objects. The age distribution is 20 years old, and 10 people are randomly selected. Among them, 1–5 are the control group, and 6–10 are the experimental group. The specific data are shown in Table 1.

### 4.3. Experimental Process

Before the experiment, it checks the results of physical fitness tests, including cardiopulmonary function, muscle strength and endurance, flexibility, body composition, and other physical fitness test results. The subjects were divided into an experimental group (*n* = 5) and a control group (*n* = 5). The experimental group conducted a 15-week sports dance intervention experiment. The control group followed the normal study and daily routine and did not do physical exercise outside the school physical education class. Cardiopulmonary function, muscle strength and endurance, flexibility, and body composition metrics were measured before and after surgery.

## 5. Experimental Results of Physical Dance Training

### 5.1. Cardiopulmonary Endurance Index

This paper selects three cardiorespiratory endurance indicators: maximal oxygen uptake, diastolic blood pressure, and systolic blood pressure to reflect the students' cardiovascular function. Among them, the unit of maximal oxygen uptake is mL/(kg·min).  Table 2 is the measurement data results of the two groups of college students in terms of cardiorespiratory endurance before and after the experiment.

As can be seen from Table 2, there was a significant difference in the maximum oxygen uptake between the control group and the experimental group after the experiment. The maximal oxygen uptake of the control group changed from 30 ± 5 to 29 ± 6, and there was no significant change. In contrast, the VO2 max in the control group increased from 29 ± 4 to 33 ± 5. The systolic blood pressure and diastolic blood pressure in the experiment were significantly different from those before the experiment. The diastolic blood pressure in the control group decreased from 75.32 ± 12.45 to 74.36 ± 11.36. The diastolic blood pressure in the experimental group decreased from 72.23 ± 10.69 to 66.02 ± 11.22. The systolic blood pressure in the control group decreased from 124.56 ± 12.56 to 122.18 ± 14.64. The systolic blood pressure in the experimental group decreased from 117.95 ± 14.23 to 112.85 ± 11.23. It shows that regular participation in physical dance has a certain effect on increasing the maximum oxygen uptake and lowering blood pressure.

### 5.2. Muscle Strength/Muscular Endurance Index

In this study, three indicators, maximal inspiratory/expiratory pressure, maximal transdiaphragmatic pressure, and maximal maintenance ventilation, were selected to evaluate muscle strength/endurance.  Table 3 shows the data changes between the experimental group and the control group before and after the experiment.

As can be seen from Table 3, there was no significant difference in the maximum inspiratory/expiratory pressure between the control group and the experimental group after the experiment. The maximum inspiratory/expiratory pressure of the control group changed from 90.9 ± 8.5 to 91.8 ± 6.6. The maximum inspiratory/expiratory pressure of the control group was 92.1 ± 7.9 and changed to 92.3 ± 4.4. The maximum transdiaphragmatic pressure and maximum maintenance ventilation in the test were significantly different from those before the test. The maximum transdiaphragmatic pressure in the control group increased from 150 ± 39 to 155 ± 40. The maximum transdiaphragmatic pressure in the experimental group increased from 147 ± 40 to 160 ± 30. The maximum maintenance ventilation in the control group increased from 90 ± 10 to 91 ± 8, and the maximum maintenance ventilation in the experimental group increased from 89 ± 6 to 96 ± 6. It shows that regular participation in physical dance has a certain effect on increasing the maximum transdiaphragmatic pressure and the maximum maintenance ventilation.

### 5.3. Flexibility Index

In this paper, 10 students were trained in physical dance for 15 weeks, including 5 in the control group and 5 in the experimental group. The effect of physical dance on flexibility was judged by observing weekly seat forward flexion. The results are shown in Figure 7.

It can be clearly seen that there is no significant difference in the index of sitting body forward flexion in the control group in the experiment. There were significant differences in the changes of sitting body forward flexion in the experimental group. It keeps increasing with the time of physical dance exercise.

### 5.4. Comprehensive Comparison of Mental Health Levels

Before the experimental intervention, each group was tested and analyzed to observe the changes in the psychological health of the experimenters, including the measurement of interpersonal relationships and self-esteem. 1 is before the experiment in the control group, 2 is after the experiment in the control group, 3 is before the experiment in the experimental group, and 4 is after the experiment in the experimental group. The results are shown in Figure 8.

After the experiment, the emotional indicators of the control group did not fluctuate much. However, the negative emotional indicators such as depression score and compulsion score of the subjects in the experimental group were significantly different from those before the experiment, and all of them were reduced to a certain extent. The interpersonal relationship score was significantly improved, which was 1.5 points higher than that before sports dance training.

### 5.5. Comparison of Subjective Well-Being Effects

Before the experiment, the subjective well-being of each group was analyzed to observe the changes in the mental health of the experimenters, including the measurement of emotion, satisfaction, and overall subjective well-being. 1 is before the experiment in the control group, 2 is after the experiment in the control group, 3 is before the experiment in the experimental group, and 4 is after the experiment in the experimental group. The result is shown in Figure 9.

As can be seen from Figure 9, there is not much difference between the control group before and after the experiment. The overall emotional scores of the subjects in the experimental group were significantly different from those before the experiment. After the experiment, the scores of the subjects in the experimental group were significantly different from those before the experiment. Happiness satisfaction increased by 7.8%.

### 5.6. Comparison of the Effect of Self-Acceptance on the Results

Before the experiment, a self-acceptance analysis was carried out for each group to observe the changes of the subjects' mental health, including measurement acceptance and evaluation acceptance. 1 is before the experiment in the control group, 2 is after the experiment in the control group, 3 is before the experiment in the experimental group, and 4 is after the experiment in the experimental group. The results are shown in Figure 10.

As can be seen from Figure 10, there is not much difference between the control group before and after the experiment. The overall emotional scores of the subjects in the experimental group were significantly different from those before the experiment. After the experiment, the self-acceptance influence total score of the experimental group was higher than that before the experiment.

### 5.7. Comparison of Self-Evaluation Effects

Before the experiment, self-evaluation was scored for each group, and it was observed whether the subjects' self-score changed before and after the experiment. Among them, 1–5 are the control group, 6–10 are the experimental group, and the self-evaluation is scored out of 100 points. The results are shown in Figure 11.

As can be seen from Figure 11, there is not much difference between the control group before and after the experiment. The self-evaluation scores of the subjects in the experimental group were significantly different from those before the experiment. After the experiment, the self-evaluation total score of the experimental group was higher than that before the experiment.

## 6. Discussion

The positive effects of dance practice on the physical and mental health of modern students after sports dance intervention are consistent with previous studies. This study found that the effect of sports dance on the physical health of modern college students is particularly obvious in improving physical fitness and muscle strength. However, interventions in dance movements have not yet had a significant impact on students' cardiorespiratory capacity, muscular endurance, and body composition. Dance movement has a major impact on the mental health of modern students. Among them, the main ones were stress, depression, sleep and nutrition, relationships, paranoia, mental health determinants, and overall performance. There were also significant improvements in the happiness index and life satisfaction factors, as well as self-acceptance and self-confidence factors in the test group.

## 7. Conclusion

Through the health examination of modern college students, this paper finds that sports dance has a positive impact on students' physical and mental health and has a greater impact on students' mental health. It has a more obvious effect on physical health by improving the cardiovascular function of college students, improving muscle strength, and improving students' flexibility indicators, especially improving body shape and muscle strength. In terms of mental health, it can help relieve students' stress and anxiety in the learning process and improve their brain quality. It promotes positive attitudes and health in students, enables them to better accept themselves, and develops the ability to improve self-correction and facilitate interpersonal face-to-face communication. At the same time, it can also improve students' self-improvement abilities and improve their self-esteem. Therefore, regular participation in the practice of sports dance is a good choice to promote the physical and mental development of students. It plays an important and critical role in the process of physical and mental development and has an important position and importance in the process of school education quality reform.

## Figures and Tables

**Figure 1:** Framework diagram of intelligent health detection and collection.

**Figure 2:** Android system architecture diagram.

**Figure 3:** Analysis of WiFi wireless transmission technology.

**Figure 4:** Gateway workflow.

**Figure 5:** Comparison between importance function samples and real ones.

**Figure 6:** Implementation process of particle filter algorithm.

**Figure 7:** Flexibility index measurements.

**Figure 8:** Comprehensive comparison of mental health levels.

**Figure 9:** Comparison of subjective well-being effects.

**Figure 10:** Comparison of self-acceptance impact results.

**Figure 11:** Comparison of self-assessment impact results.

**Table 1:** Student data collection form.

Serial number	Gender	Height (cm)	Age	Weight (kg)	Profession
1	Male	178	20	71	Preschool education
2	Female	166	20	50	Nursing
3	Female	160	21	42	Film and television
4	Female	159	21	43	Psychology
5	Male	174	19	62	Mathematic major
6	Male	183	20	75	Management
7	Female	159	20	45	Preschool education
8	Male	179	21	71	Economics
9	Male	184	22	80	Law degree
10	Female	167	20	51	Nursing

**Table 2:** The test of cardiorespiratory endurance index of subjects in the control group and the experimental group before and after the experiment.

Test indicators	Control group (*n* = 100)		Experimental (*n* = 100)	
	Before experiment	Experimental	Before experiment	Experimental
Maximal oxygen uptake	30 ± 5	29 ± 6	29 ± 4	33 ± 5
Diastolic blood pressure	75.32 ± 12.45	74.36 ± 11.36	72.23 ± 10.69	66.02 ± 11.22
Systolic blood pressure	124.56 ± 12.56	122.18 ± 14.64	117.95 ± 14.23	112.85 ± 11.23

**Table 3:** Muscle endurance index matching test of subjects in the control group and experimental group before and after the experiment.

Test indicators	Control group (*n* = 100)		Experimental (*n* = 100)	
	Before experiment	Experimental	Before experiment	Experimental
Max inspiratory/expiratory	90.9 ± 8.5	91.8 ± 6.6	92.1 ± 7.9	92.3 ± 4.4
Max transdiaphragmatic	150 ± 39	155 ± 40	147 ± 40	160 ± 30
Max maintain ventilation	90 ± 10	91 ± 8	89 ± 6	96 ± 6

## Data Availability

The data underlying the results presented in the study are available within the manuscript.
